# Improved ECG-Derived Respiration Using Empirical Wavelet Transform and Kernel Principal Component Analysis

**DOI:** 10.1155/2021/1360414

**Published:** 2021-10-15

**Authors:** Shuxin Zhuang, Fenlan Li, Zhemin Zhuang, Wenbin Rao, Alex Noel Joseph Raj, Vijayarajan Rajangam

**Affiliations:** ^1^Key Laboratory of Digital Signal and Image Processing of Guangdong Province, Shantou, Guangdong, China; ^2^Department of Electronic Engineering, Shantou University, Shantou, Guangdong, China; ^3^Centre for Healthcare Advancement, Innovation and Research, VIT, Chennai, Tamil Nadu, India

## Abstract

Many methods have been developed to derive respiration signals from electrocardiograms (ECGs). However, traditional methods have two main issues: (1) focusing on certain specific morphological characteristics and (2) not considering the nonlinear relationship between ECGs and respiration. In this paper, an improved ECG-derived respiration (EDR) based on empirical wavelet transform (EWT) and kernel principal component analysis (KPCA) is proposed. To tackle the first problem, EWT is introduced to decompose the ECG signal to extract the low-frequency part. To tackle the second issue, KPCA and preimaging are introduced to capture the nonlinear relationship between ECGs and respiration. The parameter selection of the radial basis function kernel in KPCA is also improved, ensuring accuracy and a reduction in computational cost. The correlation coefficient and amplitude square coherence coefficient are used as metrics to carry out quantitative and qualitative comparisons with three traditional EDR algorithms. The results show that the proposed method performs better than the traditional EDR algorithms in obtaining single-lead-EDR signals.

## 1. Introduction

Respiratory signals are important physiological signals commonly used in clinical monitoring. They are used in the detection of sleep apnoea and in stress tests; moreover, they play an important role in the clinical diagnosis of diseases [1]. Respiratory signal detection methods can be divided into two main categories. The first is to detect the air flow from the human nose, and the second is to detect thoracic deformation or the change in thoracic impedance caused by respiration [2]. Both methods require additional sensors and may interfere with natural breathing.

The idea of soft sensors is a one of the solutions to overcome the issues of detecting respiratory signals. Soft sensor is an inferential model that uses easily accessible variables to estimate the variables, which are difficult to be obtained. At present, soft sensors have been widely adopted in industrial processes [3]. The Luenberger observer [4] used state differential equations, with which the dynamic behaviour of the bioprocess is described with a mechanistic model. Yan et al. [5] proposed a framework of data driven soft sensor modeling based on semisupervised regression to estimate the total Kjeldahl nitrogen in a wastewater treatment process.

Obtaining respiratory signals from the ECG is a typical application of soft sensor in the medical field. The ECG signal is obtained noninvasively using a few electrodes and recorded conveniently without interfering natural breath. Respiration affects ECG signals mainly through mechanical interactions and respiratory sinus arrhythmia (RSA) [6]. Mechanical interaction is caused by the displacement of the electrodes relative to the heart and the change in thoracic impedance caused by variations in lung volume [7]. RSA is caused by breath-induced changes in the autonomic nervous system, which in turn causes changes in the heart rate. Heart rate increases during inspiration and decreases during expiration [8]. Respiration affects the heart rate and ECG in the aforementioned two ways, and such a signal modulation phenomenon forms the theoretical basis for obtaining respiratory signals from ECGs, called ECG-derived respiratory signals.

Owing to the advantages of the EDR algorithm, scientists have conducted multiple studies in this field. Most EDR methods are divided into two categories [9]. One is the EDR method based on the morphological characteristics of the ECG signal. The other is by directly processing the ECG signal. Vargas-Luna et al. [10] obtained the EDR signals through the *R* peak amplitude of ECG signals. Bailón et al. [11] proposed an EDR method based on singular value decomposition of the intervals between the *R* peaks of ECG signals. Chazal et al. [12] obtained EDR signals by calculating the area under the QRS complexes. The EDR methods are based on a single morphological characteristic that provides a rather unsatisfactory accuracy and robustness. Nemati et al. [13] proposed a data fusion method for estimating respiratory frequency based on Kalman filtering, which involves many other physiological signals, and only the respiratory rate can be obtained. Widjaja et al. [14] used kernel principal component analysis to calculate the QRS complexes in the ECG signal and considered the eigenvector as the EDR signal. This method performs well but requires manual deletion of ectopic QRS complexes that involve considerable calculations.

To resolve the limitations of the existing methods and realize an accurate and fully automatic EDR signal obtaining method, an improved EDR algorithm based on EWT and KPCA is proposed. The ECG signal is decomposed to obtain the low-frequency component. Multiple signal decomposition methods, such as wavelet approaches or empirical mode decomposition (EMD) [15], are available at present. However, the disadvantages of this method cannot be ignored. Traditional adaptive wavelet approaches often use prescribe scale subdivision scheme, which is hard to achieve an ideal adaptability. For example, the wavelet packets used a constant prescribe ratio, leading to a limited adaptability. The Brushlet method [16] decomposed the signal on Fourier spectrum, and it is also based on a prescribe subdivisions. EMD shows an ideal adaptability, but its main issue is that it lacks mathematical theory. EWT incorporates the advantages of the above two methods. It not only has rigid mathematical basis but also can decompose signal adaptively.

After using EWT to decompose the ECG signal into five modes, three modes with the lowest frequency are selected to form a new signal. Meanwhile, the *R* peak positions are determined using the Pan–Tompkins algorithm to help locating the QRS complexes. Then, the new signal is sampled based on the position of the QRS complexes. However, a few ectopic samples are captured during sampling. To address this challenge, a method based on variance is developed to delete ectopic samples automatically. Finally, to capture the nonlinear relationship between respiratory and ECG, the processed samples are processed using KPCA and preimaging to obtain the EDR signal. The radial basis function (RBF) is adopted as the kernel function of KPCA; hence, considerable calculations are required when selecting the parameters of the RBF kernel function [17]. Therefore, the parameter selection algorithm is improved in this study to reduce the calculation load.

Our contributions in this paper are as follows. (1) The EDR algorithm framework of EWT + KPCA is proposed to overcome the disadvantages of traditional EDR algorithm based on morphological characteristics of ECG signals, but also captured the nonlinear relationship between respiratory and ECG. (2) A new method based on variance to automatically delete the abnormal samples is introduced during sampling procedure. (3) The selection of RBF kernel parameters in KPCA algorithm is improved to reduce the computational requirement.

The remaining sections of this paper are organized as follows. In Section 2, the EDR algorithm based on EWT and KPCA is described in detail. In Section 3, the proposed method is compared with three traditional EDR algorithms. The qualitative and quantitative experimental results are presented. The results are discussed in Section 4, and conclusions are presented in Section 5.

## 2. Methodology

The EDR method proposed in this study is divided into two parts and shown in Figure 1. Part 1 involves the decomposition of the ECG signal based on EWT. The ECG signal is decomposed into five modes with different spectral sizes based on EWT; three modes with the lowest frequencies are selected to form a new signal. Part 2 describes the steps for obtaining the EDR signal based on the KPCA. First, the Pan–Tompkins algorithm is used to find the *R* peaks of the ECG signal, and then the QRS complexes are located. Second, the new signal formed by the three modes is sampled based on the locations of the QRS complexes, while some ectopic samples are deleted automatically. These samples serve as the input matrix for KPCA. Third, the input matrix is mapped to a higher-dimensional space through KPCA. The eigenvalues and eigenvectors of the kernel matrix are calculated. Finally, the eigenvector corresponding to the maximum eigenvalue is selected for preimaging to obtain the EDR signal.

### 2.1. Decomposition of ECG Signal Based on EWT

In general, the human respiratory rate is approximately 0.1–0.5 Hz. To extract the modes with a low-frequency ECG signal completely and adaptively, EWT is used to decompose the ECG signal. The low-frequency modes are reconstructed to form a new signal.

EWT is a mode decomposition algorithm proposed by Gilles [18]. The main concept is to extract the different modes of a signal by designing an appropriate wavelet filter bank, including a low-pass filter and several band-pass filters. The low-pass filter is used to extract the approximate component, and the band-pass filter is used to extract the component details. The number of decomposed modes is selected adaptively in the traditional EWT algorithm. Different ECG signals may be decomposed into different numbers of modes, which affects the following calculation. To unify the number of decomposed modes while ensuring the performance of EWT, the number of decomposed modes is set to five based on the experiments. The specific steps to implement the EWT algorithm are as follows:

(1) The local maxima in the spectrum of the ECG signal *f*(*t*) are obtained and sorted out in decreasing order after normalization. Next, the first six local maxima are selected, and the boundaries of each mode *ω*_*n*_(*n*=1,2,…, 5) are defined as the center of two consecutive maxima.
(2) After determining the boundaries, the empirical scaling function *φ*_*n*_(*ω*) and empirical wavelet *ϕ*_*n*_(*ω*) are constructed using the Littlewood–Paley–Meyer wavelet [19]. Here, *φ*_*n*_(*ω*) and *ϕ*_*n*_(*ω*) are expressed as
  (1) $$\begin{array}{c} \varphi_{n}\left(\omega \right)=\left\{\begin{array}{cc} \left|\omega \right|\leq \omega_{n}\left(1-\gamma \right),\\ \cos\left[\frac{\pi }{2}\beta \left(\frac{1}{2\tau_{n}}\left(\left|\omega \right|-\omega_{n}+\tau_{n}\right)\right)\right], & \left(1-\gamma \right)\leq \left|\omega \right|\leq \left(1+\gamma \right),\\ 0, & \text{otherwise,} \end{array}\right) \end{array}$$
  (2) $$\begin{array}{c} \phi_{n}\left(\omega \right)=\left\{\begin{array}{cc} \left(1+\gamma \right)\omega_{n}\leq \left|\omega \right|\leq \left(1-\gamma \right)\omega_{n+1},\\ \cos\left[\frac{\pi }{2}\beta \left(\frac{1}{2\tau_{n}}\left(\left|\omega \right|-\omega_{n+1}+\tau_{n+1}\right)\right)\right], & \left(1-\gamma \right)\omega_{n+1}\leq \left|\omega \right|\leq \left(1+\gamma \right)\omega_{n+1},\\ \sin\left[\frac{\pi }{2}\beta \left(\frac{1}{2\tau_{n}}\left(\left|\omega \right|-\omega_{n}+\tau_{n}\right)\right)\right], & \left(1-\gamma \right)\omega_{n}\leq \left|\omega \right|\leq \left(1+\gamma \right)\omega_{n},\\ 0, & \text{otherwise,} \end{array}\right) \end{array}$$
where *τ*_*n*_=*γω*_*n*_*n*(0 < *γ* < 1). Here, *β*(*x*) should satisfy the following condition:
  (3) $$\begin{array}{c} \beta \left(x\right)=\left\{\begin{array}{cc} 1 & \text{if }x\leq 0\text{ and }\beta \left(x\right)+\beta \left(1-x\right)=1\\ 0 & \text{if }x\geq 0 \end{array},\;\forall x\in \left[0,1\right].\right) \end{array}$$
Since numerical functions satisfy the above condition, we choose *β*(*x*)=*x*^4^(35 − 84*x*+70*x*^2^ − 20*x*^3^) according to [18].
(3) The different modes of *f*(*t*) are obtained by *φ*_*n*_(*ω*) and *ϕ*_*n*_(*ω*). The detail coefficient *W*_*f*_^*ε*^(*n*, *t*) and approximate coefficient *W*_*f*_^*ε*^(0, *t*) are defined as
  (4) $$\begin{array}{c} W_{f}^{\varepsilon }\left(n,t\right)=f,\psi_{1}=\int f\bar{\psi_{1}\left(\tau -t\right)}\text{d}\tau ={\left(\overset{\wedge }{f}\left(\omega \right)\bar{\psi_{n}\left(\omega \right)}\right)}^{\vee }, \end{array}$$
  (5) $$\begin{array}{c} W_{f}^{\varepsilon }\left(0,t\right)=f,\varphi_{1}=\int f\bar{\varphi_{1}\left(\tau -t\right)}\text{d}\tau ={\left(\overset{\wedge }{f}\left(\omega \right)\bar{\overset{\wedge }{\varphi_{1}}\left(\omega \right)}\right)}^{\vee }, \end{array}$$
where ∧and ∨ refer to the Fourier transform and its inverse transform. From equations (1)–(5), the empirical mode *f*_*k*_(*t*) can be obtained as
  (6) $$\begin{array}{c} f_{0}\left(t\right)=W_{f}^{\varepsilon }\left(0,t\right)*\varphi_{1}\left(t\right),\\ f_{k}\left(t\right)=W_{f}^{\varepsilon }\left(n,t\right)*\psi_{n}\left(t\right). \end{array}$$

After the three steps of processing, the ECG signal is decomposed into five modes.  Figure 2 shows the results of the time domain and frequency domain of a 10 s ECG signal after EWT.

As shown in Figure 2(b), the spectra of the five modes are sorted out in increasing order. To extract the low-frequency part of *f*(*t*) completely and adaptively, the first three modes are selected to form a new signal. The new signal *f*_*s*_(*t*) is shown in Figure 3.

Figure 3 shows that *f*_*s*_(*t*) only preserves the low-frequency part and abandons the high-frequency part of *f*(*t*), which prevents the influence of high-frequency noise on subsequent calculations. Here, *f*_*s*_(*t*) serves as the input for the following KPCA algorithm.

### 2.2. EDR Signal Acquisition Based on KPCA

KPCA is a generalization, proposed by Scholkopf et al. [20], of principal component analysis in high-dimensional feature space. In KPCA, the data are mapped to a high-dimensional feature space that is nonlinear to the input space. Using KPCA, the EDR acquisition algorithm can describe the nonlinear interaction between the ECG signals and respiratory signals. The steps of KPCA in the proposed method are described in detail in this section.

Before performing the KPCA algorithm, the input matrix *X* should be determined. The evaluation of *X* consists of the following steps:

(1) The first step is detection of *R* peaks: the positions of all the *R* peaks in *f*(*t*) are obtained using the Pan–Tompkins algorithm [21], denoted as *X*_*R*_={*x*_*i*_}_*k*=1_^*n*^. The parameter *n* is the number of *R* peaks in *f*(*t*). The Pan–Tompkins results are shown in Figure 4.
(2) The second step is sampling of the signal *f*_*s*_(*t*): after the detection of the *R* peaks, a fixed window is selected to sample the signal *f*_*s*_(*t*). In this study, *x*_*i*_ is regarded as the window center, and *f*_*s*_(*t*) is sampled in the range of 40 ms before and after *x*_*i*_. Then, the samples are used to construct the matrix *X*′ with dimensions *m* × *n*, where *m* is the length of the fixed window and *n* is the number of *R* peaks. Because the sampling interval of the ECG signal in this study is 4 ms, the value of *m* is fixed at 21.
(3) The third step is deletion of ectopic samples: as shown in Figure 5(a), there might be some ectopic samples in *X*′ that affect the accuracy of subsequent calculations. Therefore, an adaptive method based on variance is proposed to delete ectopic samples automatically. The specific steps are as follows:
  (1) First, {*α*_*i*_}_*i*=1_^*n*^ is denoted as the result of sampling, and *X*′ can be written as *X*′=[*α*_1_, *α*_2_,…, *α*_*k*_,…, *α*_*n*_]. The average sample is defined as
    (7) $$\begin{array}{c} \alpha_{\text{mean}}=\frac{1}{n}\sum_{i=1}^{n}\alpha_{i}. \end{array}$$
  (2) The matrix *Y* is defined as *Y*=[*α*_1_ − *α*_mean_,…, *α*_*k*_ − *α*_mean_,…, *a*_*n*_ − *α*_mean_], and the variance of each column vector in *Y* is calculated. The results are expressed by the vector *V*=(*v*_1_, *v*_2_,…, *v*_*k*_,…, *v*_*n*_).
  (3) It is assumed that the ectopic samples are *α*_*p*_ and the normal samples are *α*_*q*_, and in the equation, the condition, *v*_*p*_ ≫ *v*_*q*_, is satisfied. The ectopic samples are removed according to this property, and an input matrix *X* without ectopic samples is obtained.

The outline of the matrix *X* is shown in Figure 5(b).

After the input matrix *X* is determined, KPCA is introduced. The essence of KPCA is to solve the following equation:

(8) $$\begin{array}{c} \lambda v=Cv, \end{array}$$

where *λ* and *v* are the eigenvalues and eigenvectors of matrix *C*, respectively. Here, *X*=[*x*_1_, *x*_2_,…, *x*_*k*_,…*x*_*r*_], where *r* is the number of samples in *X*, and an implicit nonlinear mapping is defined as *φ*. Then, the mapped data of *x*_*k*_ in the high-dimensional feature space F can be defined as *φ*(*x*_*k*_). In equation (8), *C* is the covariance matrix of *φ*(*x*_*k*_), which is defined as

(9) $$\begin{array}{c} C=\frac{1}{n}\sum_{j=1}^{r}\varphi \left(x_{j}\right)\varphi {\left(x_{j}\right)}^{T}. \end{array}$$

Equation (8) is equivalent to the following equation:

(10) $$\begin{array}{c} \lambda \left(\varphi \left(x_{k}\right)*v\right)=\left(\varphi \left(x_{k}\right)*Cv\right),\;k=1,2,\ldots ,n. \end{array}$$

When *v*=∑_*i*=1_^*r*^*α*_*i*_*φ*(*x*_*i*_) and the RBF is introduced as the kernel function *k*(*x*, *y*),

(11) $$\begin{array}{c} k\left(x,y\right)=e^{-\left(x-y^{2}/2\sigma^{2}\right)}. \end{array}$$

After the kernel function is determined, equation (10) can be written as

(12) $$\begin{array}{c} r\lambda \alpha =K\alpha . \end{array}$$

where *α* is the vector constituted by parameter *α*_*i*_ and *K* is the kernel matrix corresponding to *k*(*x*, *y*). To extract the principal component, the projection of a test point *φ*(*x*) on the eigenvector *V*^*k* is calculated using

(13) $$\begin{array}{c} \left(v^{k}*\varphi \left(x\right)\right)=\sum_{i=1}^{r}\alpha_{i}^{k}\left(\varphi \left(x_{i}\right)\varphi \left(x\right)\right). \end{array}$$

The aforementioned computation is carried out in the high-dimensional feature space F, whereas the construction of the EDR signal is based on the first eigenvector of the input space. The eigenvalues and eigenvectors obtained in F cannot be directly used for constructing the EDR signal. To solve this problem, a limited number of eigenvectors can be used to find approximations of the data in the input space. This process is called ‘preimaging' [22]. Therefore, the first eigenvector of the input space is reconstructed by preimaging the first eigenvector of F. The EDR signal can be obtained by performing cubic spline interpolation on the reconstructed first eigenvector of the input space.

During the process of KPCA, the parameter *σ*^2^ must be carefully selected so that KPCA can deliver a better performance. First, *σ*^2^ is roughly determined as var(*z*), which is denoted as ${\hat{\sigma }}^{2}=\mathrm{var}\left(z\right)$. Parameter *z* represents the vector transformed by *X*. Then, *σ*^2^ is further tuned in the range, $\left(0,{\hat{\sigma }}^{2}\times 100\right),$ with a step of *σ*^2^/10. The steps are as follows [14]:

1. KPCA is applied to the range $\left(0,{\hat{\sigma }}^{2}\times 100\right)$ for *σ*^2^ to obtain the eigenvalues denoted as *γ*=(*γ*_1_, *γ*_2_,…, *γ*_*i*_)
2. Here, *d*=*γ*_1_ − (*γ*_2_+⋯+*γ*_*i*_) and is calculated for each *σ*^2^. Then, *σ*^2^ is selected, which achieves the maximum *d*

Although the aforementioned method can determine the appropriate *σ*^2^, it requires high computational effort because the eigenvalues of the kernel matrix are calculated for each *σ*^2^. However, *d* reaches its maximum early and decreases monotonically thereafter, as shown in Figure 6(a). Thus, the calculation of the monotonically decreasing part is redundant. Therefore, in this study, *d* is determined when the aforementioned two steps are done. When *d* reaches its maximum, the selection process of *σ*^2^ is terminated, as shown in Figure 6(b), and the *σ*^2^ corresponding to the maximum of *d* is selected for subsequent calculations.  Figure 6 shows an example of a curve graph of *d*. As shown in the figure, if not terminated at the maximum *d*, the algorithm calculates the eigenvalues of the kernel matrix 1000 times. If terminated at the maximum *d*, only 180 calculations are required. In this way, not only the accuracy of *σ*^2^ is ensured, but also the computational effort is reduced.

## 3. Results

In this section, the proposed EDR methods are compared with three traditional EDR methods, including KPCA-based [14], R-peaks-interval-based [23], and R-peaks-amplitude-based [24] EDR methods. The experimental results and the metrics of morphological similarity are presented to evaluate the performance of the aforementioned EDR methods.

### 3.1. Material

The ECG signals and reference RESP signals were provided by the Fantasia database and Shantou Institute of Ultrasonic Instruments Co., Ltd. (SIUI). The Fantasia database [25] was collected from healthy subjects in a supine posture at a sampling rate of 250 Hz.

### 3.2. Morphological Similarity Metrics

To measure quantitatively, the morphological similarity between the EDR signal and the reference respiratory signal, the correlation coefficient (C) and magnitude squared coherence coefficient (MSC) were introduced [24]. *C* is expressed as

(14) $$\begin{array}{c} C=\frac{1/\left(m-1\right)\sum_{k=1}^{m-n}\left(R_{\text{ref}}\left[k\right]-\bar{R_{\text{ref}}\left[k\right]}\right)\left(R_{\text{EDR}}\left[k+n\right]-\bar{R_{\text{EDR}}\left(k+n\right)}\right)}{\sqrt{1/{\left(m-1\right)}^{2}\sum_{k=1}^{m}{\left(R_{\text{ref}}\left[k\right]-\bar{R_{\text{ref}}\left[k\right]}\right)}^{2}\sum_{k=1}^{m}{\left(R_{\text{EDR}}\left[k\right]-\bar{R_{\text{EDR}\left[k\right]}}\right)}^{2}}}, \end{array}$$

where *m* is the length of the EDR signal and *R*_ref_ and *R*_EDR_ represent the reference RESP and EDR signals, respectively. The MSC is defined as

(15) $$\begin{array}{c} {\text{MSC}}_{xy}\left(f\right)=\frac{{\left|P_{xy}\left(f\right)\right|}^{2}}{P_{xx}\left(f\right)P_{yy}\left(f\right)}, \end{array}$$

where *P*_*xx*_(*f*) and *P*_*yy*_(*f*) represent the power spectral densities of *x* and *y*, respectively, and *P*_*xy*_ is the cross-power spectral densities of *x* and *y*. The spectra were calculated using Welch's method, a periodic Hamming window, and an overlap of 50%.

### 3.3. Experimental Results

To compare the proposed method to the three traditional EDR methods in an intuitive manner, some of the experimental results are presented in this section.

As shown in Figure 7, the EDR signal obtained by the algorithm in this study has a competitive similarity to the reference respiratory signal. As Figures 7(f) and 7(g) show, the proposed method performs well in extracting some of the RESP signals with poor quality.

Figure 8 shows that the proposed method performs better than the three traditional EDR methods. In addition, the proposed method achieves a better performance than the three traditional EDR methods in extracting poor-quality RESP signals. Figure 8(d) shows that the proposed method maintains a relatively high morphological similarity with the poor-quality RESP signals. However, the EDR signals obtained by the three traditional EDR methods differ significantly from the reference RESP signals in terms of morphology.

In addition to the aforementioned qualitative comparison results, the performances of the proposed method and three traditional EDR methods were evaluated using C and MSC.

Figure 9 shows the experimental results of the four EDR methods based on the Fantasia database and SIUI. The box plots in Figure 9 specify the median values and interquartile ranges (IQRs). As shown in Figure 8 and Table 1, the EDR methods based on a single morphology characteristic of the ECG signal (RR-interval-based and RPA-based EDR algorithm) show poor results for C and MSC; they also have the disadvantage of poor robustness. Although the KPCA-based EDR method is good, there is still a gap between it and the proposed method in terms of accuracy and robustness. In general, the proposed method is superior to the three traditional EDR methods.

To measure the performance of the proposed method for different age groups, young (21–34 years old) and elderly (68–85 years old) subjects are chosen for the experiment. The experimental results are shown in Figure 10.

As shown in different age groups, methods based on single ECG signal morphological characteristics have the disadvantages of poor robustness and low accuracy. The proposed method exhibits better performance in samples of different ages.

## 4. Discussion

### 4.1. Preprocessing

In this study, the ECG signal was decomposed into five different modes, and the three modes with low frequencies were selected to construct a new signal for EDR signal acquisition. No denoising algorithm is introduced in the proposed method. This is because the RESP signal with a relatively low frequency causes a baseline drift to the ECG signal. The correction of baseline drift by the denoising algorithm affects the extraction of the RESP signal to a certain extent. The influence of high-frequency noises is also mitigated because the three modes with lower frequency are chosen for subsequent calculation, as mentioned in Section 2.1.

### 4.2. The Effect of the Number of the Extracted Modes

In this paper, EWT is introduced to adaptively decompose the ECG signal into 5 modes, and low-frequency modes are reconstructed to form a new signal. In this section, we carried out experiments on the effect of the number of modes extracted from EWT. Here, 30 ECG signals with a length of 10 s were randomly selected and are decomposed into 4, 5, and 6 modes, respectively. C and MSC are introduced to evaluate the performance. The results are presented in Figure 11, revealing the better performance when the number of modes extracted from EWT is 5.

### 4.3. Computational Effort

In general, EDR methods involving KPCA are computationally intensive. To evaluate the extra computational effort of the proposed method with respect to the three traditional EDR methods, the computation time is recorded. Because all the mentioned EDR methods must locate the *R* peak through the Pan–Tompkins algorithm, the time required by the PTK algorithm is deducted. This experiment is based on Intel Core i7-9750H 2.60 GHz and runs on MATLAB 2018A. Five ECG signals with a length of 10 s are randomly selected from the Fantasia database for five tests. The results show that the average computation time of the proposed method and the EDR algorithm based on KPCA, *R* peaks-interval, and RPA is 0.161 s, 0.312 s, 0.006 s, and 0.013 s, respectively. The data reveal that the EDR method based on the morphological characteristics of ECG signals has a higher computational speed than the EDR method using KPCA, but at the expense of accuracy and robustness. There are two main reasons for this difference in computational complexity:

1. The EDR algorithms based on the morphological characteristics of ECG signals only process the specific characteristics (such as *R* wave amplitude and *R* wave interval) of each cardiac cycle, while the EDR algorithm using KPCA should process the entire QRS complex of each cardiac cycle. There is a huge gap in the amount of data to be processed by the two methods.
2. KPCA algorithm is complex. In addition, repeated calculation is required when choosing the parameter *δ* of RBF kernel function. It is found through experiments that in traditional KPCA-based EDR algorithm, the computational time of searching for appropriate parameter *δ* accounts for more than 90% of the total computational time of KPCA.

In the proposed method, the average computation time of the KPCA part is only 0.074 s owing to the mechanism of determining parameter *d*, whereas the average time required to compute the KPCA part in the traditional KPCA-based EDR algorithm is 0.267 s. The time saving rate reached 72.3%, which significantly reduces the computational effort.

## 5. Conclusions

The proposed EDR method based on EWT and KPCA shows good performance than the traditional EDR methods in the extraction of EDR signals from single-lead-ECG signals. The ECG signal is decomposed into five different modes through the EWT, and a new signal is formed by constructing the three components with a low frequency. Then, the new signal is sampled to form the input matrix based on the location of the QRS complex, and an ectopic sample removal method is used to delete the ectopic samples. Subsequently, KPCA is used to obtain the eigenvectors and eigenvalues. Finally, the EDR signal can be obtained by processing the results using preimaging and cubic spline interpolation. After the selection method of the parameters of the RBF kernel in KPCA is improved, the computation time is significantly reduced, alleviating the problem of high computational effort in the EDR method with KPCA to a certain extent. Experimental results show that the proposed method performs better than the three traditional EDR methods and is suitable for monitoring respiration through single-lead-ECG signals without additional sensors.

## Figures and Tables

**Figure 1:** The proposed EDR method based on EWT and KPCA.

**Figure 2:** ECG signal of 10 s in time and frequency domains: (a) ECG signal and the corresponding Fourier spectrum, in which the red dotted line in the spectrum graph is the boundary of different modes, and the green boxes represent the high-frequency noise and (b) the five modes of EWT in time and frequency domains.

**Figure 3:** Distribution of *f*_*s*_(*t*) in time and frequency domains.

**Figure 4:** Results of Pan–Tompkins algorithm (the red circles are the locations of the *R* peaks).

**Figure 5:** Outline of (a)*X*′ and (b) *X*: the abscissa is the length of the fixed window.

**Figure 6:** Curve graphs of *d*: (a) applying KPCA to the range $\left(0,{\hat{\sigma }}^{2}\times 100\right)$ without terminating at the maximum of *d* and (b) terminating at the maximum of *d*.

**Figure 7:** Comparison of the EDR signal obtained by the proposed method and the reference RESP signal. In each picture, the subplot above is the EDR signal, and the subplot below is the reference RESP signal.

**Figure 8:** Performance of the proposed method compared with those of the KPCA-based, R-peaks-interval-based (RR interval), and R-peaks-amplitude-based (RPA) EDR methods.

**Figure 9:** Comparison between the proposed method and three traditional EDR methods: (a) correlation coefficients and (b) magnitude squared coherence coefficients.

**Figure 10:** Comparison of four EDR algorithms based on ECG signals of different ages: (a, b) the results of elderly samples and (c, d) the results of young samples.

**Figure 11:** Comparison of different numbers (*N*) of the modes extracted from EWT.

**Table 1:** C, MSC, and IQR of the four EDR methods.

Method	EWT + KPCA	KPCA	RR interval	RPA
C	0.730	0.600	0.439	0.485
IQR (C)	0.685–0.808	0.706–0.498	0.6130–0.267	0.311–0.665
MSC	0.784	0.680	0.516	0.655
IQR (MSC)	0.755–0.897	0.626–0.782	0.657–0.400	0.504–0.780

## Data Availability

Part of the data used in this paper can be found in the website https://physionet.org/about/database/, and the other part is the data provided by the SIUI, which is not open to the public because it involves privacy.
